The article "Evaluating the predictive value of fetal Doppler indices and neonatal outcome in late-onset preeclampsia with severe features: a cross-sectional study in a resource-limited setting" was retracted in 2025. Reasons: errors in the analysis; unreliable results or conclusions; concerns about the data; concerns about the welfare of human subjects.

# Evaluating the predictive value of fetal Doppler indices and neonatal outcome in late-onset preeclampsia with severe features: a cross-sectional study in a resource-limited setting

**DOI:** 10.1186/s12884-022-04704-0

**Published:** 2022-05-01

**Authors:** Eman Mohamed Ibraheim Moawad, Amr Samir Fouad Tammam, Maha Mohamed Mosaad, Hadeer Mashaal El Sayed, Adel Atef

**Affiliations:** 1 Department of Pediatrics, Faculty of Medicine, Cairo University, Giza, Egypt; 2 Department of Obstetrics and Gynecology, Faculty of Medicine, Cairo University, Giza, Egypt

**Keywords:** Severe, Late onset preeclampsia, Adverse outcomes, Fetal Doppler indices

## Abstract

**Background:**

Preeclampsia constitutes a major health problem with substantial maternal and perinatal morbidity and mortality. The aim of this study was to detect the diagnostic efficacy of fetal Doppler in predicting adverse outcomes in severe late onset preeclampsia (LOP).

**Methods:**

A prospective study was conducted among childbearing women who presented with severe LOP and matched controls. Umbilical artery (UA) and middle cerebral artery (MCA) Doppler indices including pulsatility index (PI), resistance index (RI), systolic/diastolic ratio (S/D) and cerebroplacental ratio (CPR) were measured.

**Results:**

All UA indices were significantly higher in the case group compared to the controls (*p* < *0.001*). UA PI and RI were significantly correlated with all neonatal adverse outcomes except cord pH status (*p* < *0.05*). Abnormal CPR was the most sensitive index that positively correlated with intrauterine growth retardation (IUGR), low 5- minute Apgar score and neonatal intensive care unit admission (79, 72.8 and 73.3%, respectively). In the same context, Abnormal UA PI and RI represented the most specific tool for predicting IUGR, low 1- and 5- minutes Apgar score with positive predictive values were 52, 87 and 57%, respectively.

**Conclusion:**

In severe LOP, UA Doppler remains the preferential indicator for adverse birth outcomes with CPR is the best index that could be solely used for predicting such outcome.

## Background

Preeclampsia (PE) is a complex pregnancy-specific hypertensive disorder arising after 20 weeks’ gestation [1]. It constitutes a major health problem associated with substantial maternal and perinatal morbidity and mortality with increased risk of long-term health consequences [2]. The worldwide-level estimates of PE range from 3 to 10% of all pregnancies with more than 70.000 maternal mortalities and over 500.000 fetal/neonatal deaths annually [1, 3]. In low- and middle-income countries, the prevalence is rapidly increasing almost 7 times more (2.4%) than developed ones (0.4%) [3]. In 2014, a multi cross- sectional survey conducted in 29 developing countries reported that a range of 1 in 10 to 1 in 4 perinatal deaths were attributed to severe PE and eclampsia [4]. In Egypt, around 960 maternal deaths occur annually with PE identified as the main indirect cause of death [5].

Based on the onset, PE is further classified into two main types, early onset (EOP) and late onset (LOP) with cut-point of ≤ 34 weeks gestation. The latter accounts for the majority of cases (> 80%) [6]. The pathogenesis of PE is quite complex and poorly understood. However, it is believed that the main feature is urtero-placental insufficiency with compensatory changes of fetal circulation in response to hypoxia [6, 7]. These circulatory adaptations could be non-invasively detected by Doppler ultrasound waveforms [7].

In limited resource settings as in Egypt, prevention of health burden related to PE represents a major challenge. Thus, from a health and financial perspective, employing reliable non-invasive simple techniques is warranted to reduce the impact of PE arise mainly from premature birth, neonatal complications and stay in neonatal intensive care unit (NICU) [8].

Therefore, we evaluated the umbilical artery (UA) and middle cerebral artery (MCA) with cerebroplacental ratio (CPR) using different Doppler ultrasound parameters to detect its diagnostic efficacy for predicting adverse outcomes in pre-eclamptic women with severe features presented at ≥ 34 weeks of gestation.

## Methods

### Study design and context

We conducted a hospital-based prospective, cross-sectional study included a cohort of childbearing women ≥ 34 weeks of gestation with severe PE (case group) and group of matched healthy childbearing females (control group) between September 2018 and March, 2019. All study participants were recruited from Obstetrics and Gynecology Department, Kasr Al Aini Hospital that serves as a tertiary referral center for more than 220 thousand women across Egypt and Middle East region annually. The department incorporates six inpatient units, surgery, antenatal care, and fetal medicine with 297 bed capacity [9]. The sample size was obtained to yield a 95% confidence level, 5% margin of error with anticipated response rate 80%.

### Study population

All childbearing women who presented to the Labor and Delivery triage unit at Kasr Al Aini hospital during a six- month study period were screened for eligibility. The case group (Group I) was comprised of sixty women with a viable singleton pregnancy ≥ 34 weeks, complicated by LOP with severe features and delivered by caesarean section (CS) who consented to participate. All women who met eligibility criteria and had existing comorbidities (e.g., diabetes, renal disorders etc.), and those complicated by intrauterine fetal death and fetal anomalies were also excluded. A comparison group of 60 healthy, non-preeclamptic, parity-, maternal age- and gestational age- matched women with uncomplicated singleton pregnancies were recruited during the same calendar period (Group II).

### Operational definitions

Pre-eclampsia with severe features was diagnosed based on criteria set by International Society for the Study of Hypertension in Pregnancy (ISSHP) as illustrated in Table 1 [10].

**Table 1:** Diagnostic criteria of pre-eclampsia and severe pre-eclampsia [10, 11]

Preecalmpsia
Proteinuria of ≥ 0.3 g in a 24-h urine specimen, protein (mg/dL) /creatinine (mg/dl) ratio of 0.3 or higher, or a urine dipstick protein of 1
**Other maternal organ dysfunctions, including:**
Acute kidney injury (AKI) (creatinine ≥ 90 μmol/L; 1 mg/dL)
liver involvement (elevated transaminases e.g., ALT or AST > 40 IU/L) with or without right upper quadrant or epigastric abdominal pain)
Neurological complications e.g., altered mental status, blindness, stroke
Hematological complications (thrombocytopenia – platelet count below 150,000/μL, DIC, hemolysis)
Uteroplacental dysfunction e.g., fetal growth restriction
**Severe features of preeclampsia**
-Elevated blood pressure (systolic ≥ 160 mm Hg, diastolic ≥ 110 mm Hg)
-Elevated creatinine level (> 1.1 mg per dL [97 μmol per L] or ≥ 2 times baseline)
-Hepatic dysfunction (transaminase levels ≥ 2 times upper limit of normal) or right upper-quadrant or epigastric pain
-New-onset headache or visual disturbances
-Platelet count < 100 × 103 per μL (100 × 109 per L)
-Pulmonary edema

Gestational age was estimated based on maternal recall of the first day of last menstrual period (LMP) and/or the ultrasound measurement of the crown-rump length in first trimester, if available.

For purpose of this study, adverse neonatal outcomes were defined as occurrence of one or more of the following: 1- and / 5- minutes Apgar score < 7, metabolic acidosis at birth (pH < 7.20), low birth weight (LBW) (defined as birth weight of less than 2500 g) [12], intrauterine growth retardation (IUGR) (defined as fetal abdominal circumference or estimated fetal weight < 10^th^ percentile and umbilical Doppler PI > 95^th^ percentile on ultrasound scan) [13] and admission to NICU.

### Study measurements

To assure consistency and minimize interpersonal biases, all participating physicians were instructed regarding selection and exclusion criteria, definitions and procedures prior to the study. In addition, the neonatologists were evaluated in the delivery room for adequate Apgar score interpretation.

All study population were subjected to full history taking including demographic data (age, parity, and gestational age), current health status and occurrence of any chronic illnesses. Two well-trained nurses were assigned to measure the blood pressure for all study population using automated well-calibrated device validated to be used in pregnancy following guidelines for measuring blood pressure in the clinic setting. Mercury sphygmomanometer was used concurrently with respect to National Institute for Health and Care Excellence (NICE) antenatal Care guidance steps [14].

Immediately, after birth, the clinical status of newborn infants was evaluated by the attending neonatologist using Apgar score at 1 and 5 min of life. Other data included gestational age and birth weight were assessed by New Ballard scoring system [15] and Niklasson percentile growth curves, consecutively [16].

Samples for blood gas analysis were collected from pulsating unclamped umbilical cords of all neonates in sterilized heparinized syringes labelled with patient identifier. After collection, samples were immediately placed in ice and transferred to the laboratory and results were obtained within 30 min from collection.

### Doppler ultrasonography

Doppler analysis was performed for all study participants using the same ultrasound machine (SAMSUNG Model: SONOACE R3) and by the same physician (AMA) with over 10 years of antenatal Doppler ultrasound experience. Doppler indices of fetal UA and MCA were measured including:

- Pulsatility index (PI) = Peak systolic velocity – End diastolic velocity / Time-averaged maximum velocity
- Rresistance index (RI) = systolic velocity—diastolic velocity / Peak systolic velocity
- Systolic/diastolic ratio (S/D) ratio = Peak systolic velocity/End- diastolic ratio, calculated from blood flow velocities.

These Doppler indices were recorded automatically from consecutive waveforms with the angle of insinuation below 30°. The UA Doppler waveform was produced by sampling a free-floating portion of the umbilical cord using colour Doppler and UA PI, RI and S/D ratio were calculated according to the standard protocol [17]***.*** A transverse section of the fetal head was obtained, and MCA was identified, using colour Doppler, at the level of its origin from the circle of Willis. The MCA was sampled using pulsed Doppler with the vessel passing the sphenoid wing and PI, RI, S/D ratio were calculated according to the standard protocol [18]***.*** Cerebroplacental ratio is calculated by dividing the MCA PI/ UA PI (i.e., MCA S/D to UA S/D) [19].

In the current study, reference values for fetal Doppler indices were based on the study conducted by Ciobanu et al. [19]. All measured Doppler values were plotted on the appropriate reference range for the corresponding centile charts [19]. Umbilical artery, MCA and CPR indices were defined as being abnormal if values > 95^th^ percentiles, < 5^th^ percentiles and < 1, respectively.

### Data management and statistical analysis

Data were statistically described in terms of mean, standard deviation (± SD), median and range for qualitative data or frequencies (number of cases) and percentages for categorical data. Comparison of numerical variables between the study groups was done using the Student *t* test for independent samples when normally distributed and Mann Whitney *U* test for independent samples when not normally distributed. For comparing categorical data, Chi square (*χ*^2^) test was performed. When the expected frequency is < 5, Fisher’s exact test was used instead. The test of sensitivity, specificity, positive and negative predictive values (PPV and NPV) were also used. *P*-values less than 0.05 were considered statistically significant. All statistical calculations were coded and entered using the statistical package SPSS (Statistical Package for the Social Sciences) version 25.

## Results

In total, 1295 pregnant women with a mean age of 25.3 ± 7.6 (17 – 45) years were assessed for eligibility during the study period. Out of those patients, 910 participants didn’t meet inclusion criteria and 118 didn’t consent to be in the study. The recruitment pathway led to final participation of 120 patients allocated into two groups of 60, cases (Group I) and controls (Group II). (Fig. 1).

**Fig. 1:** Recruitment flowchart for study participants

Pertinent maternal and neonatal characteristics of the study participants are shown in Table 2. There was no significant difference between both groups in terms of maternal age, parity, and gestational age. The overall mean age was 29.7 (± 6.2) years with no statistical difference between both groups (*p* = *0.568*). Approximately, 65% of patients were multigravida. The study women gave birth to singleton neonates with mean gestational age was 37.1 (± 1.5) weeks at birth, ranging from 34 to 41 weeks (Table 2).

**Table 2:** Distribution of demographic, obstetric characteristics and neonatal outcomes of the study population

Variable	Group I (cases) *N* = 60	Group II (Controls) *N* = 60	Total *N* = 120	*P* value
**Age:** mean (± SD)	29.4 ± 6.3 (18- 38)	30 ± 6.1 (18- 43)	29.7 ± 6.2 (18—43)	0.568
**Parity:** n (%)				
- **Primigravida**	23 (38)	20 (33)	43 (36)	0.568
- **Multigravida**	37 (62)	40 (67)	77 (64)	
**GA at delivery in weeks:** mean (± SD)	36.9 ± 1.5 (34–41)	37.3 ± 1.5 (34—40)	37.1 ± 1.5 (34—41)	0.152
**Preterm birth:** n (%**)**	22 (36.7)	17 (28.3)	39 (32.5)	0.435
**APGAR score at:** mean (± SD)				
• 1 min	5.08 ± 1.97 (3—8)	7.6 ± 0.81 (7—9)	6.34 ± 1.95 (3—9)	** < 0.001**
• 5 min	7.18 ± 1.35 (3 – 10)	9.2 ± 0.4 (9—10)	8.19 ± 1.41 (3—10)	** < 0.001**
**Cord pH:** mean (± SD)	7.31 ± 0.08 (6.96 -7.5)	7.39 ± 0.03 (7.28 -7.45)	7.35 ± 0.07 (6.96 -7.5)	** < 0.001**
**Birth weight (grams):** mean (± SD)	2618.92 ± 655.63 (1200–4500)	3360 ± 337.37 (2850–4250)	2989.88 ± 639 (1200 -4500)	** < 0.001**
**Intra-uterine growth retardation: (IUGR) n (%)**	19 (31.7)	0 (0)		
**NICU admission: n (%)**	15 (25)	0 (0)		
**Death: n (%)**	3 (5)	0 (0)		

*GA* Gestational age, *NICU* Neonatal intensive care unit, *N* Number, *SD* Standard deviation

As shown in Table 2, there were statistically significant differences between both groups in perinatal outcome. In this context, severe preeclamptic group had significant neonatal morbidity in terms of lower 1- and 5-min Apgar scores, cord pH, birth weight, IUGR, NICU admission and neonatal death compared to the healthy controls (*p* < *0.001*) Table 2.

Table 3 demonstrates the mean Doppler indices in the study population. The mean PI, RI and S/D index of UA were significantly higher in the case group compared to the controls (*p* < *0.001*). The Doppler indices of the MCA showed no significant difference between both groups except for S/D index (*p* = *0.048*). Moreover, CPR showed significant difference between both groups with *p* value < *0.001*.

**Table 3:** Distribution of the median (± inter-quartile) of umbilical artery, middle cerebral artery and CPR indices among the study groups

Median ± IQ	Cases *N* = 60	Controls *N* = 60	*P* value
**UMA**			
● **PI**	1.02 ± 0.357	0.76 ± 0.05	** < 0.001**
● **R/I**	0.65 ± 0.12	0.56 ± 0.02	** < 0.001**
● **S/D**	3.19 ± 1	2.31 ± 0.11	** < 0.001**
**MCA**			
● **PI**	1.37 ± 0.27	1.37 ± 0.29	0.783
● **R/I**	0.75 ± 0.14	0.72 ± 0.07	0.423
● **S/D**	3.6 ± 0.84	3.50 ± 1.09	**0.048**
**CPR**	1.28 ± 0.84	1.85 ± 0.46	** < 0.001**

*CPR* Cerebroplacental ratio, *IQ* Interquartile, *MCA* Middle cerebral artery, *PI* Pulsatility index, *RI* Resistance index, *S/D* Systolic/diastolic ratio, *UA* Umbilical artery

Table 4 illustrates the correlation between fetal Doppler indices and maternal blood pressure of the study population. No statistically significant correlations were found between maternal blood pressure, either systolic or diastolic, and Doppler indices included UA, MCA, and CPR in both severe pre-eclamptic patients and healthy control groups (*p* > *0.05*) Table 4.

**Table 4:** Correlation between fetal Doppler indices (umbilical artery, middle cerebral artery and cerebro-placental ratio) with maternal systolic and diastolic blood pressure

Doppler	Index	Cases				Controls				
		**SBP**		**DBP**		**SBP**			**DBP**	
		**R**	***P* value**	**r**	***P* value**	**r**	***P* value**	**R**		***P* value**
**UA**	**PI**	- 0.127	0.333	0.060	0.651	0.030	0.820	-0.046		0.726
	**RI**	0.157	0.231	0.030	0.819	0.036	0.784	-0.067		0.609
	**S/D**	0.136	0.299	0.200	0.126	0.017	0.897	-0.105		0.425
**MCA**	**PI**	-0.03	0.821	0.102	0.439	0.024	0.853	0.042		0.752
	**RI**	0.046	0.726	-.090	0.492	-0.039	0.769	-0.078		0.555
	**S/D**	0.024	0.855	0.207	0.112	-0.021	0.876	-0.066		0.617
**CPR**		0.146	0.266	0.012	0.925	-0.070	0.593	0.021		0.876

*CPR* Cerebroplacental ratio, *DBP* Diastolic blood pressure, *MCA* Middle cerebral artery, *PI* Pulsatility index, *RI* Resistance index, *SBP* Systolic blood pressure, *S/D* Systolic/diastolic ratio, *UA* Umbilical artery

Employing Pearson coefficient among the case group didn’t reveal significant correlation between the degree of proteinuria in group I and fetal Doppler indices. For UA PI, RI and S/D ratio, correlation coefficient values were (*r* =—0.02,—0.02 and – 0.009) with *P* values (0.530, 0.130 and 0.310, respectively). As for fetal MCA PI, RI and S/D ratio, correlation coefficient values were (*r* =—*0.083,—0.198 and – 0.133* with *P* values (*0.878, 0.881 and 0.947*), respectively. The correlation between CPR and proteinuria was also insignificant (*r* =—*0.065, p* = *0.621*).

The correlation and association between fetal Doppler indices and adverse pregnancy outcomes were presented in Table 5. In terms of worse outcomes, the UA Doppler indices were statistically significantly correlated with Apgar score assessed at 1- and 5- minutes in neonates born to severely pre-eclamptic mothers (*p* < *0.05*) except for the S/D index which had no significant correlation with 5- minute Apgar score (*p* = *0.094*). Conversely, the MCA indices had no significant correlation with immediate neonatal outcomes in terms 1- and 5-min Apgar score (*p* > *0.05*). All fetal Doppler indices exhibited no statistically significant correlation with the acid–base status at birth (*p* > *0.05*). Referring to the same table, we found that PI and RI of both UA and MCA as well as CPR were statistically significantly associated with IUGR among the case group (*p* < 0.05) (Table 5). In those neonates born to severely preeclamptic mothers and admitted to NICU (*n* = 15), UA PI and RI were the only parameters displayed statistically significant association (*p* = *0.013 and 0.019, respectively*).

**Table 5:** Correlation and association between fetal Doppler indices (umbilical artery, middle cerebral artery and cerebro-placental ratio) and adverse neonatal outcome in the study cases (Group I)

	**UA**			**MCA**			**CPR**
	**PI**	**RI**	**S/D**	**PI**	**RI**	**S/D**	
**Birthweight**							
- R	- 0.428	- 0.491	-0.04	0.015	0.184	- 0.04	0.284
- *P* value	**0.001**	** < 0.001**	0.763	0.909	0.160	0.759	**0.028**
**Apgar score**							
- **1 min**							
- R	-0.310	-0.274	-0.265	0.06	0.193	-0.250	0.198
- *P* value	**0.016**	**0.034**	**0.041**	0.648	0.139	0.054	0.128
- **5 min**							
- R	-0.270	-0.341	-0.218	0.063	0.076	-0.197	0.176
- *P* value	**0.037**	**0.008**	0.094	0.631	0.565	0.132	0.18
**PH**							
- R	0.13	0.091	-0.102	0.003	0.103	0.05	-0.118-
- *P* value	0.322	0.491	0.437	0.984	0.432	0.704	0.369
**IUGR (mean ± SD)**							
- Yes (*n* = 19)	1.33 ± 0.45	0.76 ± 0.11	3.26 ± 0.66	1.27 ± 0.3	0.69 ± 0.1	3.59 ± 0.453	1 ± 0.41
- No (*n* = 41)	1 ± 0.3	0.61 ± 0.09	3.02 ± 0.634	1.43 ± 0.23	0.75 ± 0.09	3.57 ± 0.630	1.49 ± 0.4
- *P* value	**0.001**	** < 0.001**	0.192	**0.026**	**0.013**	0.905	** < 0.001**
**NICU (mean ± SD)**							
- Yes (*n* = 15)	1.31 ± 0.51	0.72 ± 0.1	3.17 ± 0.73	0.15 ± 0.29	0.72 ± 0.11	3.73 ± 0.74	1.23 ± 0.45
- No (*n* = 45)	1.03 ± 0.31	0.64 ± 0.12	3.07 ± 0.623	1.36 ± 0.25	0.74 ± 0.09	3.53 ± 0.54	1.38 ± 0.46
- *P* value	**0.013**	**0.019**	0.620	0.160	0.487	0.246	0.299

*CPR* Cerebroplacental ratio, *IUGR* Intra-uterine growth retardation, *MCA* Middle cerebral artery, *NICU* Neonatal intensive care unit, *PI* Pulsatility index, *RI* Resistance index, *SD* Standard deviation, *S/D* Systolic/diastolic ratio, *UA* Umbilical artery

Figure 2 presents the distribution of abnormal fetal Doppler values in relation to adverse birth outcomes among the case group. Considering all the Doppler indices, approximately more than half of the Group I had abnormal CPR measurements (*n* = 31, 51.7%). Abnormal CPR was the most prevalent index associated with immediate adverse neonatal outcome in the form IUGR in 80% (*n* = 15) of infants and low 1- and 5- minutes Apgar score in 58% (*n* = 25) and 72.7% (*n* = 16) of the study cases, respectively. Almost 80% (*n* = 15) of neonates admitted to NICU had also abnormal CPR detected prior to their deliveries.

**Fig. 2:** Distribution of abnormal Doppler indices in relation to adverse neonatal outcome

Table 6 showed the diagnostic efficacy of abnormal fetal Doppler indices in predicting the adverse neonatal outcomes. In the current study, CPR exhibited the most sensitive index that positively correlated with IUGR, low 5- minute Apgar score and NICU admission (79, 72.8 and 73.3%, respectively) among the study cases. The MCA PI sensitivity for detecting low Apgar score at 1 min was the highest (73.7%) with an overall diagnostic accuracy of 78.3%. In respect to UA, its indices represented the most specific tool for predicting IUGR, low 1 and 5- minutes Apgar score with PPV values were 52, 87 and 57%, respectively Table 6.

**Table 6:** Diagnostic efficacy of abnormal fetal Doppler indices (umbilical artery, middle cerebral artery and cerebro-placental ratio) in predicting adverse neonatal outcome

Abnormal Doppler indices	Sensitivity (%)	Specificity (%)	Positive predictive value (PPV) (%)	Negative predictive value (NPV) (%)	Accuracy (%)
**UA PI (> 95**^**th**^** percentile) *N* = 23**					
- IUGR	57.9	70.7	48	78	66.7
- 1- minute Apgar score	46.5	82.4	87	38	56.7
- 5- minute Apgar score	59	73	57	76	68.3
NICU Admission	60	68.9	39	84	66.7
Overall	55.85	73.57	57.75	69	64.6
**UA RI (> 95**^**th**^** percentile) *N* = 25**					
- IUGR	68.4	70.7	52	83	70
- 1- minute Apgar score	46.5	70.6	80	34	53.3
- 5- minute Apgar score	32.6	35.3	56	17	33.3
NICU Admission	60	64.4	36	83	63.3
Overall	51.875	60.25	56	54.25	54.975
**MCA PI (< 5**^**th**^** percentile) *N* = 22**					
- IUGR	52.6	70.7	46	76	65
- 1- minute Apgar score	73.7	80.5	64	87	78.3
- 5- minute Apgar score	31.6	73.2	50	79	38.3
NICU Admission	31.6	61	27	66	51.7
Overall	47.375	71.35	46.75	77	58.325
**MCA RI (< 5**^**th**^** percentile) *N* = 22**					
- IUGR	52.6	70.7	46	76	65
- 1- minute Apgar score	32.6	53	64	24	38.3
- 5- minute Apgar score	25.6	35.3	50	16	28.3
NICU Admission	14	47	40	18	23.3
Overall	31.2	51.5	50	33.5	38.725
**CPR indices (< 1) *N* = 31**					
- IUGR	79	61	48	86	66.7
- 1- minute Apgar score	58	64.7	81	38	60
- 5- minute Apgar score	72.8	60.5	52	79	65
NICU Admission	73.3	55.6	36	86	60
Overall	70.775	60.45	54.25	72.25	62.925

*CPR* Cerebroplacental ratio, *IUGR* Intra-uterine growth retardation, *MCA* Middle cerebral artery, *NICU* Neonatal intensive care unit, *PI* Pulsatility index, *RI* Resistance index, *UA* umbilical artery

## Discussion

Doppler flow ultrasound has emerged as a non-invasive tool for maternal–fetal surveillance in high-risk pregnancies and prediction of adverse-pregnancy outcomes [7]. Consistent with previous studies [20, 21], using Doppler indices for comparison between healthy pregnant females and those with severe LOP showed significant abnormalities in the mean values of all Doppler parameters except MCA PI and RI (*p* = *0.783 and 0.423, respectively*). In 2013, Lopez-Mendes et al. reported that although the general Doppler results of MCA didn’t show significant difference between preeclamptic and control groups, however, each individual parameter could be used to predict vascular alteration specific for PE [22].

Data from randomized controlled studies provided strong evidence for effectiveness of UA Doppler, particularly PI, as an informative and a prognostic tool in management of high-risk pregnancies. In PE, raised UA PI is used as a surrogate marker for increased placental vascular impedance triggered by local hypoxia phenomena resulting in increased fetal peripheral vascular resistance and placental insufficiency [23, 24]. Such fetal surveillance has been associated with notable reduction in perinatal deaths from 1.7% to 1.2% (*RR 0.71, 95% CI 0.52–0.98*) [25]. In the current study, for all fetal Doppler measurements, UA parameters were significantly associated with poor neonatal outcome in pregnancies with severe PE compared to the healthy ones (*p* < *0.001*). Moreover, combining all UA indices (PI and RI) was found to have the highest overall specificity and PPV (66.9% and 56.9, respectively) associated with worse neonatal outcomes in all domains compared to other Doppler indices. This confirms the findings of earlier studies that proved the value of UA Doppler indices in evaluating fetal growth and well-being [26, 27].

In the last 2 decades, MCA and CPR Doppler measurements have evolved and gradually become more integrated into the clinical practice [28]. Given that 80% of fetal cerebral blood carried by it, in addition of being easily accessible by ultrasound, MCA has become the gold standard vessel for assessment of fetal intracranial perfusion [29]. Consistent with other studies, we found infants with IUGR had statistically lower MCA PI and RI mean values (*p* = *0.026 and 0.013, respectively*) compared to those born appropriate-for-gestational age [30]. Conversely, no significant association was found between MCA indices and individual Apgar scores at 1- and 5- minutes in the entire study population (*p* = *0.609*). In a systematic review and meta-analysis of 35 studies testing 4025 fetuses, Morris et al. reported that abnormal MCA Doppler values have limited predictive accuracy for compromise of fetal/neonatal wellbeing [31]. Nevertheless, in terms of prediction of adverse outcomes, the findings of our study confirmed previous reports that abnormal MCA PI and RI (*n* = 22) were more specific than being sensitive in predicting IUGR, particularly the late-onset one [32]. Additionally, we found that the abnormal MCA PI values (< 5th percentile) were the best predictor for low 1-min Apgar score in the group I newborn with sensitivity and NPV of 73.2 and 87%, respectively. This agrees with previous studies confirming that MCA waveform abnormality is considered a marker for fetal hypoxia with significant risk of perinatal morbidity and mortality [32, 33].

In our study, no statistically significant association was detected between mean CPR values of group I and neonatal outcomes in terms of 1- and 5-min Apgar score, cord pH and NICU admission (*p* = *0.128, 018, 0.369 and 0.299, respectively*). Similarly, other studies reported that although CPR represents fetal adaptation to uteroplacental hypoxia [34], however, beyond the 34^th^ week of gestation, it is not significantly related to the prognosis and outcome of the pregnancy [35]. Yet, it is noteworthy to point out that these studies have investigated CPR in the setting of routine antenatal screening not in high-risk pregnancies. In the current research, CPR ≤ 10^th^ percentile represented 51.7% (*n* = 31) of group I participants and demonstrated significant positive correlation with low birth weight (*p* < *0.028*) and a strong association with IUGR (*p* < *0.001*). These results are consistent with existing research findings reported that low CPR was significantly associated with adverse perinatal outcome [36, 37]. Compared to other indices, CPR was the most sensitive indicator to predict adverse neonatal outcomes, except for 1-min Apgar score, with overall sensitivity of 70.8% and NPV of 72.3%. This finding is in consonance with the findings of Flood et al. who reported that lower CPR values have higher sensitivities and lower specificities in predicting adverse neonatal outcomes [37]. Another study found that abnormal CPR was associated with higher rate of severe PE [38]. Also, in 2010, Shahinaj et al. concluded that low CPR (< 1) is a very good predictor for adverse outcome in the fetuses of women with PE and gestational hypertension [39].

Surprisingly, no relation was found between fetal Doppler parameters and maternal SBP and DBP as well as proteinuria among the entire study population (*p* > *0.05*). These findings were consistent with the several longitudinal studies investigating the maternal hemodynamic status in LOP during which the patients have increased cardiac output while the total vascular resistance remains relatively unchanged. This could be attributed to angiogenic (e.g., placental growth factor)/anti-angiogenic factors (e.g., soluble endoglin) imbalance being milder in LOP [40]. Also, reduced production of hydrogen sulphide, a gaseous signalling molecule with vaso-relaxant properties, in LOP may be another factor implicated in such finding [40].

Preeclampsia has been widely considered as an independent risk factor that largely contributes to IUGR [41]. In the current research, the prevalence of IUGR (19%) was slightly lower than the rates previously reported by some studies [42] and higher than others [43]. In 2015, Wicaksono et al., found that LOP has no effect on the incidence of IUGR (*p* = *0.53; PR* = *1.40; 95% CI* = *0.48–4.08*) [44].This can be explained by the fact that in LOP there is no or slight alteration of spiral arteries diameter which results in placental hypoperfusion in some but not all cases [13].

Similar to other studies [45], we found that infants born to severely pre-eclamptic mothers had a significantly lower 1- and 5- minutes Apgar scores (*n* = 43, *n* = 22, respectively) compared to the control ones (*p* < *0.001*). Approximately, 35% of neonates with a compromised Apgar score (*n* = 12) at 1 min were recovered and received a score ≥ 7 at 5 min. These findings emphasize that the neonatal outcome immediately after birth is strongly influenced by both maternal condition and presence of perinatal risk factors [46].

Measurement of cord pH is the most objective tool for assessment of acid base status at birth [47]. In our study, although umbilical cord pH values were significantly lower in group I compared to the controls (*p* < *0.001*), however, only 13% (*n* = 8) of neonates whose mothers were severely pre-eclamptic had moderate to severe academia (pH < 7.2). In a cohort retrospective study conducted in Croatia, fetal acidosis represented 5.9% in a group of neonates born to women with severe LOP [48]. Another study has yielded higher results with 22% of preterm neonates for pre-eclamptic mothers had significantly low pH [49]. In the same context, no significant correlation was found between acidity of neonates for pre-eclamptic mothers and fetal Doppler waveforms of UA, MCA and CPR (*p* > *0.05*). The same finding was reported by Fardiazar et al., who found no correlation between cord blood gases and Doppler findings in pregnancies complicated by IUGR [50]. Including CS deliveries which have less tendency towards metabolic academia may be one of the factors that contributed to such difference [26]. Additionally, previous studies reported that ductus venosus, inferior vena cava and umbilical vein Doppler indices were the best predictors for acid–base status at birth. These parameters were not employed in the current research [51].

## Conclusion

In conclusion, after comparing the accuracy of different fetal Doppler parameters in LOP with severe features, UA Doppler remains the preferential indicator of choice for adverse birth outcomes. However, for individual parameters, CPR is the best index that could be solely used for predicting such outcome. We also found that although the diagnostic efficiency of MCA indices are contradictory in severe LOP, hence, it is recommended to be used along with other Doppler indices in the setting of high risk pregnancies. Further research is warranted to determine the normal values and produce local reference charts for feto-maternal Doppler indices in Egypt. Moreover, utilizing antenatal Doppler ultrasound particularly in high-risk pregnancies could be an early warning sign for timely intervention, hence, improving the perinatal outcomes.

## Data Availability

The datasets used during the current study are available from the corresponding author upon reasonable request.

## Abbreviations

CPR: Cerebroplacental Ratio
CS: Caesarean Section
DBP: Diastolic Blood Pressure
EOP: Early Onset Preeclampsia
ISSHP: International Society for The Study of Hypertension In Pregnancy
IUGR: Intrauterine Growth Retardation
LBW: Low Birth Weight
LMP: Last Menstrual Period
NICE: National Institute for Health And Care Excellence
NICU: Neonatal Intensive Care Unit
NPV: Negative Predictive Value
PE: Preeclampsia
PI: Pulsatility Index
PPV: Positive Predictive Value
RI: Resistance Index
S/D: Systolic/Diastolic Ratio
SBP: Systolic Blood Pressure
